# Antibiotic resistance's Genotypic and Phenotypic Characteristics and the Frequency of Virulence Factors in *P. aeruginosa* Isolates Isolated from Water Samples in Iran

**DOI:** 10.1155/2022/7076433

**Published:** 2022-09-30

**Authors:** Ghasem Ghorbani, Ebrahim Rahimi, Amir Shakerian

**Affiliations:** ^1^Department of Food Hygiene, Shahrekord Branch, Islamic Azad University, Shahrekord, Iran; ^2^Research Center of Nutrition and Organic Products, Shahrekord Branch, Islamic Azad University, Shahrekord, Iran

## Abstract

*Pseudomonas aeruginosa* is a pathogenic bacterium that can contaminate water. In this study, 430 water samples were evaluated for *P. aeruginosa*, antibiotic resistance, and the abundance of virulence factors. *P. aeruginosa* was isolated from 28 (6.51%) water samples. Among the types of water, well and spring water showed the highest *P. aeruginosa* with, respectively, 20 (15.6%) and 5 (8.06%) positive samples per type of samples. Drinking water and mineral water showed minor contamination with *P. aeruginosa*. The prevalence of antibiotic resistance against meropenem, imipenem, erythromycin, gentamicin, chloramphenicol, and enrofloxacin was zero. The lowest and highest prevalence of antibiotic resistance was observed in drinking water and well water, respectively. The most abundant genes encoding antibiotic resistance in the *P. aeruginosa* were *bla_TEM_*, *bla_CTX-M_*, and *bla_SHV_*. This study also showed that the most abundant virulence genes in *the Pseudomonas aeruginosa* strain isolated from water were *algD* (15 = 3.49%), *lasB* (11 = 2.56%), *toxA* (10 = 2.32%), and *exoS* (7 = 1.63%). This study suggests that water may be a source of *P. aeruginosa* and contribute to releasing resistance genes through the food chain. Cross-contamination is the water transfer process that can cause contamination with *P. aeruginosa* in water. Therefore, hygienic principles can be effective in reducing water contamination.

## 1. Introduction

According to international standards, healthy water does not contain any microbial contamination and has some characteristics: no odor, no color, clarity, and impurity. Other specifications must be considered, such as microbial contamination, toxic substances, and the absence of harmful minerals [1].

Water is the natural source of *Pseudomonas aeruginosa* (*P. aeruginosa*) [2]. *P. aeruginosa* is a gram-negative, oxidase-positive, and aerobic bacillus found in soil and water and involved in the breakdown of organic matter. It is the cause of 18-61% of hospital deaths due to nosocomial infections [3]. *Pseudomonas aeruginosa* also contains exotoxin A (*exoA*); alkaline protease (*aprA*); exoenzymes S, U, and T (*exoS*, *exoU*, and *exoT*); elastase; and sialidase. The *exoA* gene and the pathogen *exoS* are secreted by secretory system III [4–6]. Due to the importance of this microorganism in water, the Institute of Standards and Industrial Research of Iran (ISIRI) has determined a test called water quality to identify and count *P. aeruginosa* by membrane filtration method, which includes different types of water, mineral water, and swimming pool water [7].

Some studies have identified the presence of this microorganism as an indicator of surface water contamination, domestic and agricultural effluents, or human feces. According to some researchers, the primary source of *P. aeruginosa* is in the surface waters of domestic wastewater, and it is found in 90% of wastewater samples. Its concentration in surface water receiving wastewater is from 1 to 10,000 cells per 100 ml [8].

However, the intestinal transport rate for *P. aeruginosa* in humans is low, indicating that its presence in water is not necessarily due to sewage contamination. Other sources of this microorganism are agricultural soils, drainage, and municipal wastewater. *P. aeruginosa* is directly related to human activities and is reported in fecal contaminated surface waters [9].

High antibiotic resistance of *P. aeruginosa*, especially beta-lactamases including broad-spectrum cephalosporins, quinolones, chloramphenicol, and tetracycline mainly by several antibiotic resistance genes, including *bla _TEM_*, *bla _OXA_*, *bla _CTXM-1_*, and *bla _VEB_*, is coded [10, 11]. The presence of resistance genes is the main reason for antibiotic resistance in *P. aeruginosa* strains isolated from food and clinical samples. Strains isolated from water are less resistant to antibiotics than clinical specimens [12].

In recent years, with the widespread multidrug-resistant (MDR) strains in different countries, identifying resistance-related genes has become particularly important. Therefore, the present study evaluated antibiotic resistance's genotypic and phenotypic characteristics and the frequency of virulence factors in *P. aeruginosa* isolates isolated from water samples in Iran.

## 2. Materials and Methods

### 2.1. Sampling

A total of 430 water samples, including 160 drinking water, 80 mineral water, 128 healthy water, and 62 spring water samples, were collected randomly from Isfahan, Ilam, Bushehr, and Mazandaran provinces (Iran) for six months. Water samples were collected to clean glass bottles size of approximately one liter. Samples were placed below 4°C during transportation, and testing was performed immediately after receiving the samples.

### 2.2. Isolation of *P. aeruginosa* from Water Samples

To isolate *P. aeruginosa* from samples, we followed ISO-16266-2008 International Organization of Standardization [ISO] (2008) instructions. [13]. Briefly, water sample (250 ml) was filtered through a 0.45-mm membrane (Millipore Co., Billerica, MA, United States) using a portable vacuum pump (Millivac-Mini Vacuum Pump XF54, Millipore, Merck, Germany). The membrane was placed on cetrimide agar (PCA) and incubation at 37°C for 24 hours. The colonies were selected based on color and odor (green-blue pigment with a specific odor). To confirm *P. aeruginosa* species, biochemical tests such as fermentation of lactose, citrate, indole, oxidase, DNase, and hemolysis in blood agar medium were performed. Colonies containing lactose-negative, citrate-positive, indole-negative, oxidase-positive, DNase-negative, and hemolytic bacteria were selected as *Pseudomonas aeruginosa*.

### 2.3. The Antibiotic Resistance Pattern of *Pseudomonas aeruginosa* Strains

The antibiotic resistance of *P. aeruginosa* isolated from water samples was tested using the disc diffusion method (Kirby Bauer) according to the Institute of Laboratory and Clinical Standards (CLSI, 2015) instructions. *P. aeruginosa* isolates were concentrated in Müller-Hinton agar, and after incubation at 37° C for 24 hours, bacterial susceptibility or resistance to the antibiotics was determined by the growth inhibition zone. Antibiotics discs used were manufactured by BioRad company, France, and *P. aeruginosa* standard strain (ATCC 10145) was used in this experiment as a positive control.

The antibiotic discs include tetracycline (30 *μ*g/disc), chloramphenicol (30 *μ*g/disc), imipenem (30 *μ*g/disc), sulfamethoxazole (25 *μ*g/disc), gentamicin (10 *μ*g/disc), enrofloxacin (5 mg/disc), cephalothin (30 *μ*g/disc), ciprofloxacin (5 *μ*g/disc), trimethoprim (5 *μ*g/disc), ampicillin (10 units/disc), penicillin (10 *μ*g/disc), and erythromycin (15 *μ*g/disc).

### 2.4. DNA Extraction and Molecular Detection of Virulence Factors and Antibiotic Resistance Genes

DNA was extracted following the methods of Shahrokhi et al. [14]. The overnight culture of bacteria in brain heart infusion (Merck, Germany) and DNA purification genomic kit (Fermentas Germany) extracted DNA. The DNA samples were then placed at -20° C until polymerase chain reaction (PCR).

PCR technique was used to detect virulence and antibiotic resistance genes. The list of utilized primers and the conditions for the reactions are given in Table 1. Gene amplification process was done in 25 *μ*l of a mixture including 1 unit of Taq DNA Polymerase (Fermentas, Lithuania), 200 *μ*mol dNTP (Fermentas, Lithuania), 2.5 *μ*l of 10× buffer solution (Fermentas, Lithuania), 1 *μ*mol of manganese chloride (Fermentas, Lithuania) 10 picomoles of each primer, 3 *μ*l of template DNA, and 25 *μ*l of sterile distilled water. The thermal program includes the initial denaturation temperature 94°C and 6 minutes, denaturation stage temperature 94° C and 60 seconds, the annealing stage temperature 55° C for 1 minute, the extension stage temperature 72° C for 5.5 minutes, and final extension stage temperature 72° C for 5 minutes.

### 2.5. PCR Product Electrophoresis

We followed the methods of Shahrokhi et al. [14, 15]. The distilled water was used as a negative control, and *P. aeruginosa* (ATCC 10145) was used as a positive control. PCR products were electrophoresed on 2% agarose gel. The gels were stained by Ethidium Bromide (Fermentase, Germany), and DNA strips were evaluated using UV light.

### 2.6. Statistical Analysis

The percentage of contamination in different sources and products has been calculated. The differences between groups were analyzed with SPSS statistical software (version 18) using the K2 method. The significant level was determined at *p* < 0.05.

## 3. Results and Discussion

### 3.1. Isolation of *P. Aeruginosa* from Water Samples

In this study, 430 water samples were evaluated for the presence of *P. aeruginosa*. The results of contaminated samples based on culture and molecular method (PCR) are summarized in Table 2. In this study, 28 (6.51%) isolates of *Pseudomonas* by bacteriological and PCR methods from drinking water, mineral water, well water, and spring water specimens were obtained. The highest frequency of the isolates (*n* = 20; 15.6%) was recovered from well water. In addition, all the isolates were confirmed by PCR. The prevalence of *P. aeruginosa* isolates in different water samples is shown in Table 2. The contamination rate of water samples with *P. aeruginosa* was reported 28. Drinking water and mineral water showed the lowest contamination, respectively. Statistically, no significant difference was observed between the samples (*p* > 0.05).

The well water pollution rate was significantly higher than the spring water. Therefore, groundwater is better as raw water than well water. The main reason for this is that healthy water is generally drained from the pipes to the open reservoir and exposed to the air for a long time without effective protective measures [14]. The high rate of *P. aeruginosa* contamination in spring water may be due to irregular production processes during the production process, including inadequate disinfection and formation of *P. aeruginosa* biofilms in the line [15]. Therefore, producers of drinking water should pay attention to controlling and managing the production process to ensure the safety of the water.

Szita et al. [2] reported 94 contaminated samples with *P. aeruginosa* out of 160 well water samples [2]. Wei et al. [13] reported 77 cases (24.5%) of *P. aeruginosa* from mineral water and spring water samples collected in China [14]. According to previous research by Wu et al. [16], *P. aeruginosa* contamination in raw water (30.4%) and activated carbon filtered water (38.6%) was significantly higher than in raw water (3.9%) [13]. Stoler et al. [17] reported that 41% of 80 water samples were positive for *P. aeruginosa*. They did not detect any strains of *P. aeruginosa* in the final mineral water [15]. However, the pollution rate of spring water was reported to be 6.9%, which is harmful to consumers' health. Anversa et al. [18] reported 19 cases (7.6%) of *P. aeruginosa* contamination in waters in Brazil [17].

According to the guidelines for the quality of water consumption (98/83/EC), drinking water should not be positive for the prevalence of *P. aeruginosa*, and its prevalence should be systematically controlled in the final water. Water chlorination and activated carbon filter system are the essential treatment processes for drinking water and absorb organic pollutants and microbes for water treatment [16]. Activated carbon filters can be contaminated with microorganisms and the most severe problem of microbial contamination in the whole process of drinking water treatment. Therefore, drinking water manufacturers must regularly clean, disinfect, and replace activated carbon filters [18].

Our results confirmed the contamination of water samples with *P. aeruginosa*. These results are comparable to those of *P. aeruginosa* contamination in other foods. For example, Algammal et al. [19] isolated 31.57% *P. aeruginosa* from 90 fish samples in Egypt [20]. Benie et al. [21] reported the prevalence of *P. aeruginosa* in beef, fresh fish, and smoked fish at 47.8%, 33.1%, and 20%, respectively [22]. Benie et al. [23] isolated 153 multidrug-resistant strains of *Pseudomonas aeruginosa* from beef (93), fresh fish (36), and smoked fish (24) [19]. Abd-El-Maogoud et al. [24] isolated *P. aeruginosa* from 65% of frozen mackerel (33%), frozen Sarus (30%), and tilapia samples (23%) [21].

### 3.2. The Antibiotic Resistance Pattern of *Pseudomonas aeruginosa* Strains

Table 3 (a, b) summarizes the antibiotic resistance of *P. aeruginosa* strains isolated from water. The results show that the prevalence of antibiotic resistance against meropenem, imipenem, carbapenem, erythromycin, gentamicin, chloramphenicol, and enrofloxacin was reported to be zero. The prevalence of antibiotic resistance against antibiotics used in drinking water was zero. The highest antibiotic resistance was observed in well water.

*P. aeruginosa* was resistant to tetracycline, cefotaxime, chloramphenicol, imipenem, and penicillin antibiotics. Four semisensitive samples were reported against doxycycline, gentamicin, penicillin, and ampicillin antibiotics.

In Wei et al. (2020) study [13], they determined the prevalence, virulence genes, and antimicrobial resistance of P. aeruginosa in drinking water in China. All P. aeruginosa isolates were sensitive to the 14 antibiotics (ciprofloxacin, levofloxacin, ofloxacin, norfloxacin, gentamicin, tobramycin, amikacin, polymyxin B, imipenem, meropenem, aztreonam, ceftazidime, cefepime, and piperacillin/tazobactam) tested [14]. Silva et al. [25] isolated 30 *P. aeruginosa* from drinking water resistant to one or more antibiotics [23].

Differences in results may be related to different sources of samples. In this study, raw water is mainly supplied from groundwater and less exposed to external factors. These media are rarely contaminated with antibiotics, so antibiotic-resistant *P. aeruginosa* has not been observed.

The present study results are comparable to antibiotic resistance *P. aeruginosa* in other foods. For example, *P. aeruginosa* strains isolated in Egypt showed multidrug resistance (MDR) to amoxicillin, cefotaxime, tetracycline, and gentamicin [20]. Carol et al. [26] observed that *P. aeruginosa* had high resistance to amoxicillin, moderate resistance to ampicillin, ceftazidime, nitrofurantoin, and gentamicin sensitivity tobramycin, cefotaxime, methylene, ciprofloxacin, and amikacin [24]. Benie et al. [21] examined the prevalence of *P. aeruginosa* in beef, fresh fish, and smoked fish. They found that *Pseudomonas aeruginosa* strains were mainly resistant to cefepime, imipenem, ceftazidime, ciprofloxacin, and piperacillin [22].

### 3.3. The Virulence and Antibiotic Resistance Genes

This study also showed that the most abundant virulence genes in the *Pseudomonas aeruginosa* strain isolated from water were *algD* (15 = 3.49%), *lasB* (11 = 2.56%), *toxA* (10 = 2.32%), and *exoS* (7 = 1.63%). This study suggests that water may be a source of *P. aeruginosa* and contribute to releasing resistance genes through the food chain. Tables 4 and Table 5 summarize the antibiotic resistance and virulence genes of *P. aeruginosa* isolated from water samples. As can be seen, the most abundant genes encoding antibiotic resistance in *Pseudomonas aeruginosa* strains were bla*_TEM_*, bla*_CTX-M_*, and bla*_SHV_*. The most abundant virulence genes detected in *P. aeruginosa* were *algD*, *algU*, *lasB*, *toxA*, *exoS*, *exoT*, and *apr*.

Shi et al. [27], using the UP-MPCR method, identified five enterotoxin genes including *ExoU*, *ExoS*, *phzM*, *toxA*, and *lasB* in *P. aeruginosa* isolated from 214 drinking water and environmental isolates [25]. Wei et al. [13] identified the virulence genes *ExoU*, *ExoS*, *phzM*, *toxA*, and *lasB* from mineral water and spring water samples collected in China [14]. Wu et al. [16] identified three virulence genes, *lasB*, *phzM*, *toxA*, *ExoU*, and *ExoS*, widely distributed among *P. aeruginosa* [13]. According to previous research, *ExoU* and *ExoS* viruses have not been detected in identical isolates [6]. *P. aeruginosa* pathogenesis is closely related to the virulence genes *ExoU*, *ExoS*, *phzM*, *toxA*, and *lasB* [26, 27]. The presence of virulence genes in this study is comparable to the results of *P. aeruginosa* contamination in other foods such as fish and beef [19, 20].

### 3.4. PCR Product Electrophoresis

Figures 1–6 show the PCR product electrophoresis of *P. aeruginosa* isolated from water samples.

## 4. Conclusion

*Pseudomonas aeruginosa* is an important pathogen and a significant threat to the microbial safety of drinking water. Isolation of *P. aeruginosa* strains from water is essential because it is a potentially pathogenic bacterium for humans and indicates food quality. This study showed the prevalence of *P. aeruginosa* in well water. Due to the abundance of *P. aeruginosa* in water, especially well water and spring water, special attention should be paid to water treatment methods that will not contribute to the selection of antibiotic-resistant *P. aeruginosa*. In addition, characterization of isolates using molecular techniques can help to develop effective and accurate prevention and control measures against *P. aeruginosa* contamination of the whole drinking water production process.

## Figures and Tables

**Figure 1:** PCR product electrophoresis of 275 bp, *algD* gene (lanes 1–3: positive samples, lane 4: positive control, lane 5: negative control, lane 6: 100 bp gene ruler).

**Figure 2:** PCR product electrophoresis of 284 bp *lasB* gene and *exoS* 444 bp (lanes 1–3: positive samples 286 bp, 4 positive control, lane 284: *lasB* gene, lane 5: positive sample 444 bp sample *exoS*, lane M: 100 bp gene ruler).

**Figure 3:** PCR product electrophoresis of 270 bp *toxA* gene and 875 bp *phzM* (from left, lanes 1–3: positive samples of 875 bp *phzM* gene; lanes 4 and 5: positive sample of 270 bp *toxA* gene; lane 6: negative controls; lane 6: 100 bp gene ruler).

**Figure 4:** PCR product electrophoresis of 410 bp *algU* gene (from left, lanes 1–4: positive samples, lane 4: positive control, lane 5: negative control, lane 6: 100 bp gene ruler).

**Figure 5:** PCR product electrophoresis of 392 bp of *phzI* gene (from left, lane M: 100 bp gene ruler, lane 1: negative control, lanes 2–4: positive samples).

**Figure 6:** PCR product electrophoresis of 593 bp *bla_CTX-M_* gene and 642 bp *bla_VEB_* (from left, lane 1: negative control; lanes 2 and 3: positive samples of 593 bp *bla_CTX-M_* bp; lanes 4 and 5: positive samples, 642 bp sample *bla_VEB_* gene; lane 6: positive control; lane M: 100 pb gene ruler).

**Table 1:** List of primers used to detect virulence factors in *P. aeruginosa* strains isolated from water [28].

Virulence genes	Sequence (5′–3′)	Size of product (bp)
*algD*	F: AAGGCGGAAATGCCATCTCC R: AGGGAAGTTCCGGGCGTTTG	275
*algU*	F: CGCGAACCGCACCATCGCTC R: GCCGCACGTCACGAGC	410
*lasB*	F: ACACAATACATATCAACTTCGC R: AGTGTGTTTAGAATGGTGATC	284
*toxA*	F: ATGTGCAGYACCAGTAARGT R: TGGGTRAARTARGTSACCAGA	270
*plcH*	F: CACACGGAAGGTTAATTCTGA R: CGGTTARACGGCTGAACCTG	608
*plcN*	F: CGACTTCCATTTCCCGATGC R: GGACTCTGCAACAAATACGC	481
*exoS*	F: GTGTGCTTTATGCCATGAG R: GGTTTCCTTTTCCAGGTC	444
*exoT*	F: CATCGTCTACGCCATGAG R: AGCAGCACCTCGGAATAG	1159
*exoY*	F: GGAATGAACGAAGCGTTCTCCGAC R: TGGCGTCGACGAACACCTCG	1035
*exoU*	F: CTGCGCGGGTCTATGTGCC R: GATGCTGGACGGGTCGAG	3308
*apr*	F: GCACGTGGTCATCCTGATGC R: TCCGTAGGCGTCGACGTAC	1017
*phzII*	F: TCCGTTATCGCAACCAGCCCTACG R: TCGCTGTCGAGCAGGTCGAAC	1036
*phzM*	F: CGTCGTGTTCAAGCAGATGGTGCTG R: CCGAACCGCTTCACCAGGC	875
*phzS*	F: CAATCATCTCAGCAGAACCC R: TGTCGTAGAGGATCTCCTG	1752
*phzI*	F: TATCGACGGTCATCGTCAGGT R: TTGATGCACTCGACCAGCAAG	392
*phzH*	F: GATTCCATCACAGGCTCG R: CTAGCAATGGCACTAATCG	1752
*lasA*	F: TGTCCAGCAATTCTCTTGC R: CGTTTTCCACGGTGACC	1075
*pvdA*	F: GCCAAGGTTTGTTGTCGG R: CGCATTGACGATATGGAAC	1281
*pilA*	F: ATGGAGAGCGGGATCGACAG R: ATGCGGGTTTCCATCGGCAG	1675
*pilB*	F: TCGCCATGACCGATACGCTC R: ACAACCTGAGCCAGCCTTCC	408

**Table 2:** The prevalence of *P. aeruginosa* in water.

Sample	*N*. samples collected	Bacteriological methods	PCR
		N. samples positive (%)	N. samples positive (%)
Drinking water	160	1 (0.6)	1 (0.6)
Mineral water	80	2 (2.5)	2 (2. 5)
Well water	128	20 (15.6)	20 (15.6)
Spring water	62	5 (8.06)	5 (8.06)
Total	430	28 (6.51)	28 (6.51)

No significant difference was observed between samples (*p* > 0.05).

**(a):** 

Antibiotic	Drinking water	Mineral water	Spring water	Well water
Tetracycline	0	1	1	1
Doxycycline	0	0	0	0
Erythromycin	0	0	0	0
Enrofloxacin	0	0	0	0
Chloramphenicol	0	0	0	0
Cephalothin	0	0	1	1
Imipenem	0	0	0	0
Carbapenem	0	0	0	0
Gentamicin	0	0	0	0
Ciprofloxacin	0	0	1	1
Trimethoprim	0	1	0	0
Sulfamethoxazole	0	0	1	1
Penicillin	0	0	0	0
Ampicillin	0	0	0	0

**(b):** 

Antibiotic	Sensitive	Semisensitive	Resistant	Total
Tetracycline	0	4	3	7
Doxycycline	6	1	0	7
Erythromycin	4	3	0	7
Enrofloxacin	4	3	0	7
Chloramphenicol	7	0	0	7
Cephalothin	4	2	1	7
Imipenem	7	0	0	7
Carbapenem	7	0	0	7
Gentamicin	7	0	0	7
Ciprofloxacin	6	0	1	7
Trimethoprim	6	1	0	7
Sulfamethoxazole	5	0	2	7
Penicillin	4	3	0	7
Ampicillin	5	2	0	7

**Table 4:** Resistance factors of *Pseudomonas aeruginosa* isolated from water.

Antibiotic resistant gene	Drinking water	Mineral water	Spring water	Well water
*bla*_TEM_	0	0	0	5
*bla*_SHV_	0	0	0	1
*bla*_OXA_	0	0	0	1
*bla*_CTX-M_	0	0	0	3
*bla*_DHA_	0	0	0	0
*bla*_VEB_	0	0	0	0

**Table 5:** Virulence factors of *Pseudomonas aeruginosa* isolated from water.

Virulence factors	Drinking water	Mineral water	Spring water	Well water
*algD*	1	1	2	11
*algU*	0	1	1	1
*lasB*	0	1	2	8
*toxA*	1	1	1	7
*plcH*	0	0	0	0
*plcN*	0	0	0	0
*exoS*	0	1	2	4
*exoT*	1	1	1	2
*exoY*	0	0	0	2
*exoU*	0	0	0	2
*apr*	0	1	1	3
*phzII*	0	0	0	0
*phzM*	0	0	1	2
*phzS*	0	0	0	0
*phzI*	0	0	0	0
*phzH*	0	1	1	1
*lasA*	0	1	1	2
*pvdA*	0	0	0	0

## Data Availability

The data that support the findings of this study are available on request from the corresponding author.
